# Taguchi-Assisted Optimization Technique and Density Functional Theory for Green Synthesis of a Novel Cu-MOF Derived From Caffeic Acid and Its Anticancerious Activities

**DOI:** 10.3389/fchem.2021.722990

**Published:** 2021-11-26

**Authors:** Malihe Zeraati, Ali Mohammadi, Somayeh Vafaei, Narendra Pal Singh Chauhan, Ghasem Sargazi

**Affiliations:** ^1^ Department of Materials Engineering, Shahid Bahonar University of Kerman, Kerman, Iran; ^2^ Department of Genetics, Islamic Azad University of Marand, Marand, Iran; ^3^ Department of Stem Cells and Developmental Biology, ACECR, Cell Science Research Center, Royan Institute for Stem Cell Biology and Technology, Tehran, Iran; ^4^ Department of Chemistry, Faculty of Science, Bhupal Nobles’ University, Udaipur, India; ^5^ Noncommunicable Diseases Research Center, Bam University of Medical Sciences, Bam, Iran

**Keywords:** Cu-MOF, anticancer, Satureja hortensis, green synthesis, lignin

## Abstract

In this paper, we have reported an innovative greener method for developing copper-metal organic frameworks (Cu-MOFs) using caffeic acid (CA) as a linker extracted from *Satureja hortensis* using ultrasonic bath. The density functional theory is used to discuss the Cu-MOF-binding reaction mechanism. In order to achieve a discrepancy between the energy levels of the interactive precursor orbitals, the molecules have been optimized using the B3LYP/6–31G method. The Taguchi method was used to optimize the key parameters for the synthesis of Cu-MOF. FT-IR, XRD, nitrogen adsorption, and SEM analyses are used to characterize it. The adsorption/desorption and SEM analyses suggested that Cu-MOF has a larger surface area of 284.94 m^2^/g with high porosity. Cu-MOF has shown anticancer activities against the human breast cancer (MDA-MB-468) cell lines, and it could be a potent candidate for clinical applications.

## Introduction

Metal-organic frameworks (MOFs) are porous adjustable crystalline polymers of three-dimensional networks of organic linkers and metal clusters. Their unique micro- or mesoporous structure results in low density, high porosity, specific surface area, and structural diversity making them attractive candidates for sensing gas, drug delivery, analysis, sensing, and energy storage (Wang et al., 2020; Zhang et al., 2021; Zhu et al., 2022). Processing and handling of MOFs are of great importance due to their crystalline nature and powder structure (Denny et al., 2016; Song et al., 2019). Many types of MOFs with different properties and porosities may be used for metal clusters, organic bonds, and inorganic minerals (Andirova et al., 2016). One way to extend the use of these functional materials is to produce MOFs on or in different media for the production of usable and cost-effective materials. Thus, MOFs are deposited or grown using direct mixing (Duan et al., 2019), *in situ* growth (Centrone et al., 2010), and layered (Lu et al., 2018) and continuous flow synthesis on different polymeric substrates, resulting in composite materials that form a complex multilevel network of microporous, mesoporous, and nanoporous, in which large and field structures increase the release kinetics and access to active fluids in microporous MOF (Mitchell et al., 2013; Marti et al., 2017). As mentioned above, MOFs have different properties, one of the most important of which is their antibacterial properties. Therefore, this application is based on the type of metal and the presence of metal ions in organic frameworks that easily enter the bacterial cell wall and alter the protein synthesis (Clearfield, 1998; Beg et al., 2017). Among different kinds of MOFs, those with open metal sites such as Al (Dhakshinamoorthy et al., 2017), Co(II) and Zn(II) (He et al., 2018), Mn (Rambabu et al., 2017), Fe (Bezverkhyy et al., 2016), Cd(II) (Ugale et al., 2017), and Cu (Yousefian and Rafiee, 2020; Zhang et al., 2020) exhibit considerable adsorption capacity for H_2_, CO_2_, CH_4_, and especially N_2_. It is worth noting that the true nature of the active sites in many MOFs, including metal ions, is saturated with the coordination of organic ligands (Zou et al., 2007). Copper has more antibacterial and anticancer properties than others (Gu et al., 2017; Pires et al., 2020). The bactericidal mechanism of Cu-MOF is due to the diffusion of Cu^2+^ ions. Also, these positive ions are absorbed by the negatively charged lipoproteins in the bacterial cell wall, enter the cell and damage the cell wall, alter its enzymatic function, or create holes in the cell wall (Abbasloo et al., 2018).

Volatile organic solvents have many environmental consequences. Green Chemistry has a wide range of solutions to reduce this problem, including short-term green reactions, but with little return (Schlesinger et al., 2010). The aromatic plant of Satureja species is used for the recovery of essential oils through hydrodistillation as well as many medicinal properties such as S. hortensis (antiproliferative activity on cancer cells), S*. khuzestanica* (antioxidant properties), and *S. montana* (antitumor activities). *Satureja hortensis* (S.H.) belongs to the family Lamiaceae and the genus *Satureja. S. hortensis* is an endemic plant that grows in tropical regions, especially in Iran, Syria, Iraq, Pakistan, and Turkey (Fierascu et al., 2018). There have been numerous studies on the biological constituents derived from lignin of these species having antibacterial and anticancer properties (Rakhmawati et al., 2009). Various studies have been performed on the extracts of S.H. extracts which show that they include caffeic acid (CA), rosmarinus acid, naringenin, isoferulic acid, and apigenin (Moghadam et al., 2015; Boroja et al., 2018). Several studies have shown that CA is the major contributor and is also known for its antioxidant potential (Moghadam et al., 2015; Mašković et al., 2017; Boroja et al., 2018; Chua et al., 2018; Fierascu et al., 2018). The use of novel organic material with several acid compounds requires optimizing the conditions of the synthesis in order to identify and investigate the effective parameters using a number of statistical methods. As a result, the Taguchi approach is one of the well-known methods for the design of experiment (DOE) (Shafiee et al., 2019a; Shafiee et al., 2019b). Simulation is also carried out to investigate the mechanism of the Cu-MOF synthesis. The density functional theory (DFT) (Shao et al., 2020) and its combination in software packages, along with methods for solving vibration modes and its intensity, have been remarkably improved in terms of hardware efficiency over the past two decades.

Taking into account the various applications of the metal organic framework (MOF) in environmental and biological aspects, the preparation of these advanced materials through the use of eco-friendly, fast, and low-cost techniques is a hot issue. It is pressing demand to prepare MOF using the fundamental concept of green chemistry. In this study, a greener method for the preparation of Cu-MOF using CuNO_3_ as a metal precursor and CA as linker has been proposed. The amount of extract, temperature, and duration of synthesis were studied by Taguchi to increase the level and efficiency of the extract, and the main mechanisms of synthesis were performed by DFT using the Gaussian-09 quantum chemistry package (Yang et al., 2021). It is characterized by FT-IR, XRD, SEM, and nitrogen adsorption and adsorption analysis. Anticancer activity is also being investigated against the human breast cancer (MDA-MB-468) cell line.

## Experimental and method

### Preparing the S.H. extract

Fresh S.H. leaves were picked from Kerman, Iran, in summer 2017. S.H. was washed with DI water and dried in the air at room temperature. Then, 100 g of the dried leaves was powdered and placed in the Clevenger-type apparatus with 1,000 ml of DI water and boiled for 60 min. The solutions were cooled and filtered by Whatman filter paper no. 1, and proteins were removed from the extract using a centrifuge at 3,000 rpm for 15 min, then stored in a dark bottle at room temperature until the solution has been used.

### Separation of CA in aqueous extract of S.H.

The Markham method has been used to extract flavonoids (Wang et al., 2021). Primarily, 250 ml of 2% AlCl_3_·6H_2_O solution was mixed with 40 ml S.H. aqueous extract. After storage for 15 min at room temperature, the powder contains CA preparations.

### Synthesis of Cu-MOF

Copper (II) nitrate trihydrate (Cu(NO_3_)_2_ 3H_2_O) (Mw 169.80 g/mol, 99.8% purity) and caffeic acid extracted from S.H. were dissolved in DI to achieve final concentrations of 0.036 M (solution A) and 0.012 M 112 (solution B). After vigorously stirring both solutions for 1 h, 30 ml of solutions A and B were combined in a glass beaker. The solution was solvothermally processed in a convective oven at 115°C for 18 h after being sonicated for 15 min. The solution was then cooled to room temperature before being centrifuged for 15 min to collect the Cu-MOF crystals. The proposed structures (1 or 2) of Cu-MOF are depicted in Scheme 1. The Cu-MOF preparation was investigated by considering the time, temperature, reactant ratio, and feed rate of the extract to the Cu precursor solution as the design parameters of the Taguchi method.

**SCHEME 1:** Proposed structures (1 and 2) of Cu-MOF.

### Taguchi method

The Taguchi method, first developed by Genichi Taguchi, is an optimization method designed to minimize the time and cost of the experiment (Yen and Lin, 2016). This method uses orthogonal arrays to organize the parameters more effectively and determine the levels of parameter change. Since the Taguchi method is classified as a fractional factorial design method, fewer experiments are needed to achieve similar results as against the complete factorial design (Zolfaghari et al., 2011; Pirzadeh et al., 2020). In the Taguchi method, different experimental conditions are tested in an orthogonal array with the aim of reducing experimental errors and process changes, enhancing process efficiency, and optimizing the set of dominant parameters (Esfandiari et al., 2018). Signal-to-noise (S/N) ratio analysis is crucial for finding optimal conditions. Smaller-better, larger-better, and nominal are the three best common types of S/N ratios for optimization that are larger and have a better algorithm according to Eq. (1) (Phadke, 1995) since a higher adsorbent selection than N_2_ is desirable.

$$S/N=\;-10\times \log\left(\overset{n}{\underset{i=1}{\sum }}{\left(\frac{1}{y_{i}}\right)}^{2}/n\right),$$ (1)

where n represents the number of replicates in the same experimental condition, and y_i_ is obtained for the target value in each experiment. Table 1 summarizes the details of each experiment. It is worth noting the numbers of trials using the Taguchi design. Minitab software was used to design the test matrix and variance analysis (ANOVA).

**TABLE 1:** Selected controlling factors and their level.

Controlling factors	Levels			
	1	2	3	4
Reactant ratio (extract/CuNO_3_)	1	1.5	2	2.5
Temperature (°C)	65	75	85	95
Time of reaction (min)	65	75	85	95
Feed rate (ml/min)	1	2	3	4

### DFT method

The DFT method obtained the molecular orbital energy of copper and S.H. extract precursors. These molecules were optimized at the theoretical level of B3LYP/3-61G as the basis for a single configuration (Mammino, 2015). All calculations were performed using Gaussian-09 (Barone et al., 2009). The optimized structures of Cu(NO_3_)_2_ precursors and CA as organic precursors molecules with their highest occupied molecular orbitals (HOMOs) and the lowest unauthorized molecular circuits (LUMOs) derived from GaussView (Shakiba et al., 2019) are shown in Figure 1.

**FIGURE 1:** Optimized structure of Cu(NO_3_)_2_ and CA precursors along with their HOMO and LUMO.

### Characterization

X-ray diffraction (XRD) was employed for the characterization and determination of the crystalline structure and phases during the synthesis of Cu-MOF. To achieve this aim, a powder X-ray diffractometer (X’PERT MPD, Malvern Panalytical, Malvern, UK; CuKα = 0.154.6 nm) was used in the range of 2θ = 4°–30° with the step width of 0.05°. A scanning electron microscope (SEM, model EM 3200, KYKY Corporation, Beijing, China) was utilized for investigation of the surface morphology. Furrier transform infrared (FT-IR; Shimadzu FT8400 spectrometer) with a Bruker Tensor 27 series was utilized for determination of vibrational frequency of the prepared samples in the range of 500 to 4,000 cm^−1^. The porosities, surface area, and pore textural characteristics of samples were determined by adsorption/desorption measures (BET, BELSORP mini II) at 77 K in an N_2_ atmosphere.

The human breast cancer (MDA-MB-468) cell line was provided by the Iranian Biological Resource Center (IBRC, Tehran, Iran). Dulbecco’s modified Eagle’s medium (DMEM), fetal bovine serum (FBS), phosphate-buffered saline (PBS), trypsin/EDTA solution, 3-(4,5-dimetylthiazol-2-Yl)-2,5-diphenyltetrazolium bromide (MTT), and dimethyl sulfoxide (DMSO) were purchased from Gibco BRL and Sigma, respectively. They were cultured in DMEM (Gibco, UK) supplemented with 10% FBS (Gibco) and 1% penicillin–streptomycin (Gibco) and incubated in a 5% CO_2_ atmosphere at 37°C. For treatment, first 5  ×  10^3^ cells per well were seeded in 96-well flat-bottomed plates overnight; second, cells were exposed to various concentrations of herbal extract (0–100 μM) and Cu-MOF (0–100 μM) for 24 and 48 h. Subsequently, the medium was removed and 200 μl of MTT solution (5 mg/ml in PBS) was added to each well and incubated for 4 h at 37°C. After discarding the solution, 100 μl of DMSO was added and the plates were shaken for 15 min. The absorbance of each sample was read at 570 nm using an ELISA microplate reader. The outcomes were affirmed as percentage of cell viability with respect to untreated control cells (Marti et al., 2017).

## Results and discussion

Table 2 shows 16 independent experiments designed using the Taguchi method and the S/N ratio associated with each experiment. All samples were analyzed with BET, and the surface area of samples was calculated. Each experiment was also repeated twice and used to calculate S/N Sabbath using Equation 1. By subtracting the maximum S/N ratio from its minimum value across the four levels, the importance of each control factor can be determined. The factor that has the least difference in the S/N ratio has less role in controlling the synthesis process (Khare and Kumar, 2012).

**TABLE 2:** The experimental design with computed selectivity and their corresponding S/N ratios.

No.	Controlling factors				BET surface area (m^2^/g)	S/N ratios
	Reactant ratio (extract/CuNO_3_)	Time of reaction (min)	Temperature (°C)	Feed rate (ml/min)		
1	1	65	45	1	946	59.51
2	1	75	60	2	302	49.6
3	1	85	75	3	220	46.84
4	1	95	90	4	859	52.88
5	1.5	65	60	3	441	58.67
6	1.5	75	45	4	12.04	54.88
7	1.5	85	90	1	1,204	10.75
8	1.5	95	75	2	555	21.61
9	2	65	75	4	1,172	61.37
10	2	75	90	3	33	45.34
11	2	85	45	2	1,642	30.37
12	2	95	60	1	2,416	64.3
13	2.5	65	90	2	2,322	67.31
14	2.5	75	75	1	1,965	65.86
15	2.5	85	60	4	185	66.44
16	2.5	95	45	3	2,100	67.66

It is concluded as shown in Table 3 that the effect of the reaction ratio (extract to CuNO3) is more significant than those of other factors. The importance of control factors can be stated in ascending order: Temperature < Reactant ratio < Feed rate < Time of reaction.

**TABLE 3:** Calculated S/N ratios and the contribution of each controlling factor.

Level	Reactant ratio (extract/CuNO3)	Temperature (°C)	Time of reaction (min)	Feed rate (ml/min)
1	33.66	40.28	32.97	43.66
2	27.75	21.86	33.87	39.03
3	35.93	34.53	37.25	29.14
4	41.24	41.92	34.49	26.75
Delta	13.49	20.06	4.27	16.91

Figure 2 shows the S/N ratio against each of the controlling factors, which are the optimal conditions for the synthesis of Cu-MOF, as follows: the reactant ratio (extract/CuNO_3_) was 2.5, the feed rate 1 ml/min, the temperature 85°C, and the time of reaction 90 min.

**FIGURE 2:** **(A)** Average value of the S/N ratio and **(B)** mean at four levels for each parameter.

The mechanism and reactivity of CA with Cu(NO_3_)_2_ precursors are defined as the energy difference of the HOMO precursor copper with LUMO acid as well as the LUMO copper with HOMO acid, shown in Figure 3.

**FIGURE 3:** The HOMO and LUMO energy levels of Cu(NO_3_)_2_ and CA.

To verify this, Cu-MOF powder was prepared with reactant CA to CuNO_3_ of 2.5, feed rate of 2 ml/min, temperature of 55°C, and time of reaction of 75-min condition which were analyzed by FTIR. The FTIR spectrum of Cu-MOF is shown in Figure 4. The broad band at 3,358 cm^−1^ is attributed to O–H stretching present in Cu-MOF, which is hydrogen bonded with surface water (Lin et al., 2015; Kaur et al., 2019). The peaks from 2,355 to 2099 cm^−1^ and 1,632 cm^−1^ are attributed to the C=O vibration in Cu-MOF (Rambabu et al., 2017) and COO as CA vibration in Cu-MOF (da Silva et al., 2015), respectively. The strong absorption peaks at 1,095, 1,152, and 1,632 cm^−1^ correspond to the C–O tensile, asymmetric, and symmetric C=O types (Lin et al., 2014; Azad et al., 2016). Adsorption bands between 872 and 995 cm^−1^ can react with symmetric and asymmetric O and C tensile vibrations of C–O of CA benzenes and react in the acid form (Stehfest et al., 2004; Liu et al., 2016). The peaks observed between 451 and 616 are assigned as vibrations inside and outside the plane of aromatic ring vibration (Stehfest et al., 2004; Mai et al., 2017).

**FIGURE 4:** Typical FTIR spectrum of Cu-MOF.

Figure 5 shows the results of nitrogen adsorption/desorption showing the porous structure of Cu-MOF at 77K. Figure 5 shows the type (I) isotherms of the IUPAC classification as an example of microporous materials (Rouquerol et al., 2013). In the early isotherm, the dramatic increase and high N_2_ uptake indicate a large proportion of microporous materials. Also, the amount of micro/mesoporous materials is very low because the isotherms of the samples in the high-pressure region do not show evidence of hysteresis and tail (Javanbakht et al., 2019). The nitrogen adsorption/desorption isotherms calculated were also related to textural parameters. The surface area measurement for Cu-MOF with BET analysis was 284.94 m^2^/g. As a result, the nitrogen uptake by Cu-MOF determines the high surface area and porosity of the sample.

**FIGURE 5:** BET isotherm of the Cu-MOF at 77 K.

Figure 6 shows that the SEM analysis was used to examine the green Cu-MOF morphology. Cu-MOF was of spherical or octahedral morphology and has a relatively uniform distribution, and the average particle size distribution is less than 100 nm (Kaur et al., 2019). Therefore, the anticancer properties of the sample were investigated. Figure 7 shows the phase formation and purity of the samples by XRD. The sample pattern belongs to Cu-MOF, the peaks marked with a circle at 31°, 37°, 43°, 52°, 59°, and 77° for Cu-MOF (JCPDS01-072-0075) (Süsse, 1967; Riccò et al., 2018).

**FIGURE 6:** SEM image of the Cu-MOF.

**FIGURE 7:** The X-ray diffraction pattern of Cu-MOF.

The cytotoxicity of copper and RA was tested *in vitro* using an MTT assay (Figure 8). The MDA-MB-468 cells were treated with different concentrations (0–100 μg/ml) of Cu-MOFs. Also, the IC_50_ values (minimum concentration of extract for reduction of the cell viability to 50%) of extracts of herbs and Cu-MOFs after incubation for 24 and 48 h were determined. The inhibitory effect of the alcoholic extract on cell proliferation was significantly higher than that of the aqueous extract. A parallel treatment of the normal cells with these components has shown a much less inhibitory effect on the viability of human normal cells (Sun et al., 2021). Firstly, up to 100 μg/ml of RA and RA-Cu shown after 24 and 48 h of incubation does not change the proliferation of MCF10-A cells, i.e., normal cells. The main property of cancer cells is uncontrolled proliferation; therefore, the control of tumor growth is considered to be a valid treatment for cancer therapy. Several studies have shown that the MOFs have beneficial aspects, including low cytotoxicity, host–guest interactions, hydrophobic/hydrophilic balance, biodegradability, body distribution, tissue accumulation, and excitability, so that such cancer treatment can be used in biological applications (Chowdhuri et al., 2017; Pathak et al., 2019; Pan et al., 2020; Niu et al., 2021). Therefore, we have chosen one type of Cu-MOF as the carrier for the antiproliferative herbal extract. Cu-MOFs appear to be more effective against the spread of breast cancer cells compared to herbal extraction. In addition, the low concentration of these biostructures (30 ± 1.2 μM) significantly reduced the growth of MDA-MB-468 cells after 48 h. As a safe anticancer agent against human breast cancer, Cu-MOF is therefore a potent component to be further explored for its cytotoxic properties.

**FIGURE 8:** Cytotoxicity of various concentrations of herbal extraction and Ag-MOF (0–100 μM) against human breast cancer cells after incubation for 24 and 48 h **(A, B)**.

## Conclusion

Cu-MOF was prepared using copper and CA as linker extracted from S.H. using ultrasonication. It has been characterized by FT-IR, XRD, SEM, and adsorption/desorption analysis, and its reaction mechanism was explained using DFT. The SEM and adsorption/desorption analyses suggested that it is extremely porous and has a large surface area of 284.94 m^2^/g. The Taguchi method was employed to optimize key parameters affecting the synthesis of Cu-MOF. It has shown excellent anticancer activities against the human breast cancer (MDA-MB-468) cell lines and could be a promising candidate as an anticancer agent.

## Data Availability

The raw data supporting the conclusion of this article will be made available by the authors, without undue reservation.
